RETRACTED

# Investigating the relationship between erythropoiesis-stimulating agents and mortality in hemodialysis patients: A systematic review and meta-analysis

**DOI:** 10.1371/journal.pone.0293980

**Published:** 2023-11-09

**Authors:** Zahra Karimi, Hadi Raeisi Shahraki, Abdollah Mohammadian-Hafshejani

**Affiliations:** 1 M.Sc. of Epidemiology, Student Research Committee, Shahrekord University of Medical Sciences, Shahrekord, Iran; 2 Assistant Professor of Biostatistics, Department of Epidemiology and Biostatistics, School of Health, Shahrekord University of Medical Sciences, Shahrekord, Iran; 3 Assistant Professor of Epidemiology, Modeling in Health Research Center, Shahrekord University of Medical Sciences, Shahrekord, Iran; University of Verona: Universita degli Studi di Verona, ITALY

## Abstract

**Background:**

In recent years, various studies have been conducted to investigate the relationship between erythropoiesis-stimulating agents (ESAs) and mortality in hemodialysis patients, who showed contradictory results. Therefore, this study aimed to investigate the relationship between ESAs and mortality in hemodialysis patients.

**Methods:**

The current study is a systematic review and meta-analysis based on observational and interventional studies published in the Web of Science, Cochrane Library, Science Direct, PubMed, Scopus, and Google Scholar databases between 1980 and the end of 2022. Jadad scale checklist and Newcastle Ottawa scale were used to evaluate the quality of articles. The study data were analyzed using Stata 15 software.

**Results:**

In the initial search, 3933 articles were extracted, and by screening and considering the research criteria, 68 studies were finally included in the meta-analysis. According to the meta-analysis results, the risk ratio (RR) of overall mortality in hemodialysis patients receiving ESAs was equal to 1.19 (95% CI: 1.16–1.23, P ≤ 0.001). The RR of mortality in patients aged 60 years and under was equal to 1.33 (1.15–1.55, P ≤ 0.001), in the age group over 60 years was equal to 1.13 (1.10–1.16, P ≤ 0.001), in randomized clinical trial studies was equal to 1.06 (0.80–1.40, P = 0.701), in cohort studies was equal to 1.20 (1.16–1.25, P ≤ 0.001), in American countries was equal to 1.19 (1.10–1.29, P ≤ 0.001), in Asian countries was equal to 1.15 (1.10–1.19, P ≤ 0.001), and in European countries was equal to 1.18 (1.05–1.34, P = 0.007).

**Conclusion:**

The results of the study show that receiving ESAs is associated with a 19% increase in the risk of overall mortality in hemodialysis patients.

## Introduction

Chronic kidney disease (CKD) is a major health challenge in the world [1]. CKD is a stage of the disease in which kidney function reaches less than 50% of its normal capacity [2]. If the kidneys are unable to function at more than 10–15% of their normal capacity, it is considered an end-stage renal disease (ESRD). At this stage, kidney transplant or hemodialysis, or peritoneal dialysis becomes necessary for survival [2, 3]. On average, worldwide, the number of patients who receive hemodialysis treatment increases by 7% annually [4]. Although the history of dialysis dates back to 1960 and since then many successes have been achieved in the treatment of these patients, their survival rate is still far lower than the survival rate of normal people in society [5].

RETRACTED

In recent years, erythropoiesis-stimulating agents (ESAs) have been widely used as a treatment for anemia in patients with CKD and patients with ESRD [6, 7]. In patients with chronic kidney failure who are treated with hemodialysis, a statistically significant relationship has been observed between anemia and low survival in these patients [7–10]. However, although the treatment of anemia leads to an increase in the survival rate in these patients, it was observed in the randomized clinical trials (RCTs) that the correction of the hemoglobin (Hb) level to the normal range in these patients using ESAs, does not lead to additional benefits [6, 7]. Therefore, concerns arose about whether the higher dose of ESA was contributing to increased mortality in hemodialysis patients. In recent years, several studies have examined the relationship between ESAs intake and mortality in hemodialysis patients [6, 11–24], however, the same results have not been observed in these studies, as in some of these studies, it has been observed that ESAs intake has a protective role against mortality in hemodialysis patients [16–18], while in other studies, a significant statistical relationship has been observed between ESAs intake and increased mortality risk [6, 11–15], in other studies, significant relationship between ESAs intake and mortality in hemodialysis patients hasn’t been observed [19–24].

Since there are no clear results in this field and one of the best ways to answer a scientific question in this medical condition is to use a systematic review and meta-analysis method, therefore the purpose of designing and implementing this study is to investigate the relationship between receiving ESAs and mortality in hemodialysis patients using the method of systematic review and meta-analysis. It can be stated that this study is the most comprehensive and complete analysis in the field of determining the relationship between receiving ESAs and mortality in hemodialysis patients to date because more recent studies and therefore more participants have been considered, so this study has provided a more convincing conclusion.

RETRACTED

## Material and methods

### Type of study and studied population

This research is a systematic review and meta-analysis using information and data from observational and interventional studies that investigated the relationship between receiving ESAs and mortality in hemodialysis patients in different regions of the world until the end of 2022.

### Search strategies

This research followed the Preferred Reporting Items for Systematic Review and Meta-Analysis (PRISMA) guidelines. A comprehensive literature search was conducted in databases including Web of Science, Cochrane Library, ScienceDirect, PubMed, Scopus, and Google Scholar for articles published through the end of 2022. The search utilized the keywords "mortality," "hemodialysis," "erythropoietin," and associated synonyms based on Medical Subject Headings (MeSH).

### Inclusion and exclusion criteria of study

This study included all clinical trials, case-control studies, cross-sectional studies, and cohort studies that examined the association between ESA use and mortality in hemodialysis patients. No restrictions were placed on time or location. Only English-language studies in human subjects that assessed the relationship between ESA use and mortality in hemodialysis patients and reported effect sizes with relative risk or odds ratio and 95% confidence intervals (CIs) were included. Exclusion criteria were lack of access to the full text after contacting the authors, as well as posters, review articles, letters to the editor, and qualitative studies.

### Specifications of study data collection tool

After collecting articles, bibliographic information and abstracts were entered into Endnote version 8 and duplicates were removed using this software and by rechecking article titles. Next, titles were screened for relevance to the research purpose; irrelevant articles were excluded. The remaining abstracts and full texts were reviewed to ensure relevance to the study purpose; any irrelevant items were removed. To increase credibility, two independent researchers (the first and third authors) completed the search and selection process. Any disagreements were resolved by the third researcher (second author) to reach consensus on final article selection. To ensure access to all relevant published research, reference lists of final articles were reviewed to identify additional related studies. For articles without publicly available full texts, the corresponding authors were contacted by email to request full texts.

Final included articles were catalogued in an Excel form with the following information: article details (title, first author, publication year, country, study design, sample size), participant characteristics (mean age, gender), intervention and control details (number of exposed and unexposed groups, patient follow-up period, ESA medication status), effect size of the ESA-mortality relationship (relative risk or odds ratio with 95% CI), and list of adjusted confounders.

RETRACTED

### Evaluation of the quality of the articles

The Jadad scale assessed the quality of RCTs. The Jadad scale scores range from 0 to 8. Studies with scores <4 considered low quality, 4–6 medium quality, and ≥7 high quality [25, 26].

The Newcastle-Ottawa Scale (NOS) assessed observational study quality (cohort, case-control, cross-sectional). NOS scores range from 0 (weakest) to 10 (strongest). Studies with scores <5 were considered low quality, 5–8 medium quality, and ≥9 high quality [27].

### Statistical methods

Due to the low incidence of the outcome under study (mortality), the estimated OR in various studies was considered as an estimate of RR [28]. In studies where the effect size was calculated and presented separately for time or seasonal periods, using the meta-analysis method, a total effect size was calculated from the presented values and considered in the analysis. Also, in studies where the effect size was not reported, but information about exposure and outcome was available, the effect size and the relevant 95% CI were estimated and considered in the meta-analysis. The presence of heterogeneity in the studies included in the meta-analysis was assessed using statistical tests (chi-square test and I2 (to report a quantitative amount of heterogeneity)) and graphical methods (forest plot). Using the Chi-square test, the differences in the results of the studies entered in the meta-analysis were investigated and the results of this test determined the type of model (fixed or random). To determine the factors related to heterogeneity in the results, the met-regression model was used by considering variables such as study sample size, article quality evaluation score, study design (randomized controlled clinical trial, case-control, or cohort studies), the average age of participants, follow-up period, the sex ratio of study participants, place of study, and the year of the study. Sensitivity analysis was also used to evaluate the effect of omitting each of the studies on the final result. Funnel diagrams and Begg’s and Egger’s tests were used to assess publication bias. Metatarium command was used to estimate the effect size of the relation in the missing studies. All analyzes were performed by Stata statistical software (version 15.0, Stata Corp, College Station, TX), and the significance level in this study was considered <0.05.

RETRACTED

## Results

According to Fig 1, 3933 articles were collected by electronically searching the databases using the keywords in Mesh and mentioning Title/Abstract. By repetition, 1056 articles were removed and 2877 articles remained. By examining each title and abstract of the articles, 2798 articles were removed because of non-English language, review articles, meetings, letter to the editor, in vivo and in vitro studies, and 79 relevant articles remained in the study. By re-examining the studies, 5 articles were found due to not reporting the effect size, 3 articles due to not reporting the confidence interval of effect size, and 7 articles because the target group included peritoneal dialysis patients in addition to hemodialysis patients, were excluded from the study and 64 articles remained in the study. Finally, by checking the list of references of these articles, 4 related articles were extracted from the references mentioned in these articles, and 68 articles were considered in the current systematic review and meta-analysis (Fig 1).

**Fig 1:** Flowchart of selected studies for meta-analysis to investigate the relationship between receiving ESAs and mortality in hemodialysis patients.

### Features of selected studies

In total, 68 studies were retrieved to investigate the relationship between receiving ESAs and mortality in hemodialysis patients. The sample size of the studies included in the meta-analysis was equal to 1,857,386 participants. The characteristics of the studies included in the meta-analysis are shown in Table 1. In terms of the geographical distribution of studies, 14 studies were conducted in Europe with a statistical population of 17,654 participants, 27 studies were conducted in America with a statistical population of 1,575,106 participants, and 27 studies were conducted in Asia with a statistical population of 264,626 participants. Of the total studies, 62 studies were performed with a cohort design, 5 studies with an RCTs design, and 1 study with a cross-sectional design (Tables 1 and 2). The prevalence of underlying diseases in the study population in each of the studies included in the meta-analysis can be seen in S1 Table in S1 File.

**Table 1:** Characteristics of the studies included in the meta-analysis to investigate the relationship between receiving ESAs and mortality in hemodialysis patients.

Number	Authors	Year	Study design	Study setting	Sample size	RR	95% CI	mean follow-up (Months)	Quality score
1	J. Bahlmann [29]	1991	randomized clinical trial	German	129	1.05	0.74–14.89	6	8*
2	J. Möcks [19]	2000	cohort	German	3111	0.81	0.51–1.37	12	8
3	Dennis J. Cotter [30]	2004	cohort	US	31301	1.67	1.35–2.06	12	10
4	HAROLD I. FELDMAN [31]	2004	cohort	US	27280	1.02	0.86–1.22	6	9
5	Deborah L. Regidor [11]	2006	cohort	US	58058	1.23	1.14–1.33	24	7
6	Brian D. Bradbury [16]	2008	cohort	US	22955	0.93	0.92–0.95	12	10
7	Elani Streja [32]	2008	cohort	US	32418	1.59	1.54–1.65	3	9
8	Ryan D. Kilpatrick [33]	2008	randomized clinical trial	US	321	0.69	0.47–1.01	12	8*
9	Chang-Chyi Jenq [34]	2009	cohort	Taiwan	187	1.014	1.002–1.026	12	8
10	Yi Zhang [21]	2009	cohort	US	18454	1.01	0.87–1.17	9	10
11	Huan-Cheng Chang [35]	2009	cohort	Taiwan	702	2.07	1.58–2.63	46.08	10
12	Brian D. Bradbury [20]	2009	cohort	US	6133	0.9	0.79–1.02	6	9
13	Joseph M. Messana [36]	2009	Cross-sectional	US	393967	1.43	1.25–1.63	-	8
14	Victor E Pollak [37]	2009	cohort	US	1774	1.41	1.19–1.66	6	9
15	Ouhong Wang [38]	2010	cohort	US	27791	1.18	1.02–1.36	12	10
16	Joan Fort [10]	2010	cohort	Spanish	2310	0.76	0.64–0.9	24	10
17	Joanne H. Lau [39]	2010	randomized clinical trial	Canada	154	1.12	1.01–1.24	72	7*
18	M. Alan Brookhart [17]	2010	cohort	US	269717	0.96	0.95–0.98	12	9
19	Alexander Kainz [40]	2010	cohort	Austrian	932	2	1.47–2.72	48	10
20	Paulo Roberto SANTOS [41]	2011	cohort	Brazil	156	5.172	1.663–16.081	12	10
21	Yi Zhang [42]	2011	cohort	US	35593	1.17	1.05–1.3	9	7
22	Eric D. Weinhandl [43]	2011	cohort	US	137918	1.07	0.96–1.18	36	7
23	Vincenzo Panichi [44]	2011	cohort	Italy	753	1.62	1.18–2.23	36	9
24	Uyen Duong [45]	2012	cohort	US	139103	1.56	1.09–2.22	22.83	9
25	Shingo Fukuma [46]	2012	cohort	Japan	95460	1.56	1.22–1.99	12	10
26	Xavier Cuevas [47]	2012	cohort	Spanish	2310	1.15	0.98–1.36	24	10
27	Anuja Shah [48]	2012	cohort	US	2402	0.74	0.59–0.91	26.26	9
28	Tetsuya Fujikawa [12]	2013	cohort	Japan	2104	2.33	1.33–4.07	27.45	9
29	Junichi Ishigami [49]	2013	cohort	Japan	349	2.73	1.2–6.24	24	10
30	Angie Nishio [50]	2013	cohort	US	606	1.85	1.44–2.4	30	8
31	Wei Yang [22]	2013	cohort	US	409 364	0.98	0.89–1.08	22.7	8
32	Marit M Suttorp [51]	2013	cohort	Netherland	1013	1.27	1.08–1.49	60	10
33	Ben C. Wong [52]	2013	cohort	Canada	484	1.6	0.76–3.61	3	9
34	Nadiesda A. Costa [53]	2013	cohort	US	36450	1.89	1.67–2.15	6	9
35	Andreas Schneider [54]	2013	randomized clinical trial	German	1015	1.77	1.23–2.54	48	8*
36	Tetsuya Ogawa [55]	2014	cohort	Japan	320	1.86	1.25–2.57	70.4	9
37	Andreas Schneider [56]	2014	cohort	German	1255	1.25	1.18–1.32	48	9
38	Masayuki Okazaki [57]	2014	cohort	Japan	248	4.204	1.173–15.065	24	9
39	Takahiro Kuragano [58]	2014	cohort	Japan	1095	1.71	0.48–6.07	24	7
40	Vincenzo Panichi [59]	2014	cohort	Italy	753	1.01	1.006–1.025	84	9
41	Owen Kwon [60]	2015	cohort	Korea	1276	1.81	1.1–2.98	19.4	10
42	Rieko Eriguchi [61]	2015	cohort	Japan	2905	1.41	1.18–1.69	48	8
43	Myoung Nam Bae [62]	2015	cohort	Korea	1594	1.72	1.1–2.68	40	10
44	Masayuki Okazaki [63]	2015	cohort	Japan	298	1.9	0.92–3.93	34.6	10
45	Kunitoshi Iseki [64]	2015	cohort	Japan	1525	0.899	0.49–1.648	36	8
46	Elani Streja [14]	2016	cohort	US	128598	1.2	1.05–1.37	60	10
47	Jiacong Luo [65]	2016	cohort	US	98972	1.64	1.39–1.94	21	9
48	Shunji Shiohira [66]	2016	cohort	Japan	375	3.64	2.03–6.28	36	9
49	Scott Sibbel [67]	2016	cohort	US	99294	0.94	0.76–1.18	12	8
50	Zijin Chen [13]	2016	cohort	China	250	2.22	1.18–4.17	36	8
51	Rafael Perez-Garcıa [18]	2017	cohort	Spanish	1679	1.47	1.11–1.94	27.7	8
52	Valeria Saglimbene [23]	2017	randomized clinical trial	Italy	656	0.98	0.64–1.52	12	7*
53	Javier Varas [68]	2017	cohort	Spanish	1679	1.97	0.75–5.14	17.79	9
54	Nada Dimkovic [69]	2017	cohort	US	603	1.225	0.704–2.129	12	8
55	Ko-Lin Kuo [24]	2018	cohort	Taiwan	42 230	0.99	0.94–1.05	41	10
56	Toshihide Hayashi [70]	2019	cohort	Japan	108	2.25	1.25–4.06	37.2	9
57	Ling Sun [71]	2019	cohort	China	159	1.112	1.029–1.202	24	9
58	Angelo Karaboyas [72]	2019	cohort	US	4604	1.06	0.88–1.29	8	10
59	Shu-Ching Yeh [73]	2019	cohort	Taiwan	1346	0.76	0.35–1.65	37	10
60	Xiangxue Lu [74]	2020	cohort	China	276	1.781	1.091–2.91	55	10
61	Sai Pan [15]	2021	cohort	China	824	1.62	1.26–2.08	12	9
62	Kenichi Tanaka [75]	2021	cohort	Japan	127	2.57	1.05–6.27	55.2	10
63	Takahiro Yajima [76]	2021	cohort	Japan	180	1.06	1.03–1.08	55.2	10
64	Yukio Maruyama [77]	2021	cohort	Japan	149308	1.025	1.021–1.029	12	10
65	Marisa Roldao [78]	2022	cohort	Portugal	59	5.4	1.31–22.32	3	10
66	Hideki Fujii [79]	2022	cohort	Japan	3312	1.42	1.1–1.84	24	10
67	Hyang Yun Lee [80]	2022	cohort	Korea	123	4.4	1.2–16.1	24	10
68	Shizuka Kobayashi [81]	2022	cohort	Japan	175	5.51	1.71–17.78	24	10

*Jadad scale

RETRACTED

**Table 2:** Adjusted variables to investigate the relationship between receiving ESAs and the mortality of hemodialysis patients in the articles included in the study.

Number	Publication first author	Year	Adjusted variables
1	J. Bahlmann [29]	1991	-
2	J. Möcks [19]	2000	-
3	Dennis J. Cotter [30]	2004	Age, sex, race, primary diagnosis, and comorbidities.
4	HAROLD I. FELDMAN [31]	2004	Iron, gender, race, age, Duration of ESRD, diabetic status, hospitalizations, IV antibiotic doses administered, URR, Albumin, AST/SGOT, Bicarbonate, Ferritin, Hemoglobin and Phosphate.
5	Deborah L. Regidor [11]	2006	-
6	Brian D. Bradbury [16]	2008	Age, sex, race, body mass index, region, diabetes status, dialysis vintage, urea reduction ratio, systolic and diastolic blood pressure, albumin level, calcium level, ferritin level, Hb level, phosphorus level, parathyroid hormone level, transferrin saturation, number of hospitalizations, number of hospitalization days, number of unexcused missed dialysis visits, number of EPO dose changes, and percentage of time with Hb level less than 11 g/dL (⬍110 g/L).
7	Elani Streja [32]	2008	-
8	Ryan D. Kilpatrick [33]	2008	Age, gender, race, diabetes mellitus, and dialysis vintage
9	Chang-Chyi Jenq [34]	2009	-
10	Yi Zhang [21]	2009	Age, race, gender, underlying cause of ESRD, geographic region, Charlson index score, cardiovascular and non-cardiovascular comorbidities, baseline hematocrit, average intravenous iron administered inpatient stays in the baseline, and average epoetin dosage and number of administrations at baseline
11	Huan-Cheng Chang [35]	2009	Age, chronic glomerulonephritis and etiology, and Fe or vitamin D3
12	Brian D. Bradbury [20]	2009	Age, race, gender, body mass index, diabetes, vascular access type, albumin, ferritin, Mean hemoglobin, transferrin saturation, systolic and diastolic blood pressure, missed EPO administrations, iron dose, and hospitalizations
13	Joseph M. Messana [36]	2009	Demographic, anthropometric, and Medicare claims data, EPO, iron, and vitamin D analogues
14	Victor E Pollak [37]	2009	age, major co-morbid conditions, IV iron, Hb, TSAT, Serum ferritin, Serum albumin, Kt/V
15	Ouhong Wang [38]	2010	Hemoglobin level and epoetin alfa dose 2, 4, 6, and 8 wk before exposure, days in the hospital, number of epoetin alfa doses administered outside the hospital, albumin, ferritin, TSAT, vascular access type, hypertension, and dialysis adequacy 2 wk before exposure.
16	Joan Fort [10]	2010	Age, functional status, body mass index, albumin levels, catheter as vascular access, and previous history of cardiovascular disease
17	Joanne H. Lau [39]	2010	Age, DM, CAD, pulse pressure, gender, average Hgb, and serum albumin
18	M. Alan Brookhart [17]	2010	Race, age, sex, geographic region indicator variables, body mass index, serum albumin, calendar year, cause of end-stage renal disease, history of ischemic heart disease, and history of stroke
19	Alexander Kainz [40]	2010	-
20	Paulo Roberto SANTOS [41]	2011	Age, high-grade comorbidity, and mean hemoglobin
21	Yi Zhang [42]	2011	-
22	Eric D. Weinhandl [43]	2011	-
23	Vincenzo Panichi [44]	2011	Age, albumin, CVD, and CRP
24	Uyen Duong [45]	2012	Age, gender, race/ethnicity, ten pre-existing comorbid conditions, history of tobacco smoking, categories of dialysis vintage, primary insurance, marital status, presence of diabetes, serum ferritin and iron saturation, body mass index, serum levels of albumin, total iron-binding capacity, creatinine, phosphorus, calcium, bicarbonate, blood white blood cell count and lymphocyte percentage.
25	Shingo Fukuma [46]	2012	Age, sex, time on dialysis therapy, post-dialysis body weight, diabetes, history of cardiovascular disease, serum albumin level, and transferrin saturation.
26	Xavier Cuevas [47]	2012	Gender, alcohol consumption, nephrologist follow-up time, CKD etiology, previous cardiac arrhythmia, SBP before HD session, hemodialysis technique, HD intolerance, glucose, phosphorus, hemoglobin, potassium, AST, phosphorus binder drugs, cardiovascular drugs, and vitamin D analogs/metabolites.
27	Anuja Shah [48]	2012	hemoglobin categories and change of hemoglobin categories and entry calendar quarter plus age, gender, presence of diabetes, race/ethnicity (African Americans and other self-categorized Blacks, Non-Hispanic Caucasians, Asians, Hispanics, and others), categories of dialysis vintage (<6 months, 6–12 months, 12–24 months, and _2 years), primary insurance (Medicare, Medicaid, and others), and marital status (married, single, divorced, and widowed), type of vascular access (catheter, AVF, and graft), dialysis dose as indicated by Kt/V (single pool), 10 preexisting comorbid conditions, history of tobacco smoking.
28	Tetsuya Fujikawa [12]	2013	Age, PCR, albumin, CRP, and phosphorus. Sex, ferritin, and comorbidities
29	Junichi Ishigami [49]	2013	Dialysis period, age, sex, Diabetes mellitus, serum albumin, serum CRP and serum ferritin
30	Angie Nishio [50]	2013	Age, sex, race, comorbidities, dialysis vintage (years on dialysis), type of vascular access, use of renin angiotensin blockers, serum albumin and Kt/V
31	Wei Yang [22]	2013	-
32	Marit M Suttorp [51]	2013	Age, sex, weight, primary kidney disease, diabetes mellitus, malignancy, cardiovascular disease. 2 Additional adjusted for weekly Kt/V urea, GFR, nutritional status, albumin, ferritin, PTH, and CRP.
33	Ben C. Wong [52]	2013	-
34	Nadiesda A. Costa [53]	2013	Age, gender, weight, race/ethnicity, hemodialysis vintage, hemodialysis catheter, diabetes status, and donor type.
35	Andreas Schneider [54]	2013	
36	Tetsuya Ogawa [55]	2014	Age, sex, dialysis vintage, body mass index, and serum albumin
37	Andreas Schneider [56]	2014	Age, sex, Atorvastatin, and 25 (OH) D.
38	Masayuki Okazaki [57]	2014	Age and serum levels of albumin and CRP
39	Takahiro Kuragano [58]	2014	-
40	Vincenzo Panichi [59]	2014	Age, dialectic vintage, Charlson index, GNRI quartiles, nPCR, and CRP
41	Owen Kwon [60]	2015	Age, sex, dialysis vintage, diabetes, cardiovascular disease, albumin, high-sensitivity C-reactive protein and ferritin and adjusted transferrin saturation (TSAT)
42	Rieko Eriguchi [61]	2015	Age, sex, dialysis duration, pre-dialysis systolic blood pressure, antihypertensive agent use, diabetes, history of cardiovascular disease, serum albumin, serum calcium, serum phosphorus, serum total cholesterol, log-transformed serum C-reactive protein, log-transformed serum ferritin, body mass index, and Kt/V
43	Myoung Nam Bae [62]	2015	Age, gender, diabetes mellitus, previous cardiovascular disease history, duration of dialysis, serum level of iron, ferritin, albumin, intact PTH, hs-CRP, total cholesterol, and Kt/V.
44	Masayuki Okazaki [63]	2015	Age, gender, geriatric nutritional index, diabetes, diastolic BP, protein catabolic rate, and Ferritin
45	Kunitoshi Iseki [64]	2015	JESS, Elderly group, Vintage, male gender, primary disease, comorbidities, congestive heart failure cancer, hypertension, neurologic disorder, CVD, BMI, Albumin, Dialysis time, Dialysis frequency, Single pool Kt/V, and Hypnotic agent
46	Elani Streja [14]	2016	Age, sex, race/ethnicity (Caucasian, African American, Hispanic, Asian, and others), marital status (married, divorced, single, and widowed), primary insurance (Medicare, Medicaid, private insurance, and others), comorbid conditions, calendar quarter of cohort entry, and dialysis vintage (<6months, 6monthsto <24 months, 2to <5years, and ≥5 years), diabetes mellitus, hypertension, ischemic heart disease, congestive heart failure, cerebrovascular disease, peripheral vascular disease, chronic obstructive pulmonary disease, malignancy, non-ambulatory state, and current smoking status, Hb level, serum albumin, creatinine, calcium, phosphorus, bicarbonate, total iron binding capacity, ferritin, white blood cell count, lymphocyte percentage, normalized protein nitrogen appearance (a metric of dietary protein intake), dialysis adequacy (single-pool *Kt/V*), and body mass index
47	Jiacong Luo [65]	2016	Age, sex, cause of end-stage renal disease, dialysis vintage, vascular access, cancer, cerebrovascular disease, heart failure, chronic obstructive pulmonary disease, coronary artery disease, gastrointestinal bleeding, human immunodeficiency virus/AIDS, peripheral vascular disease, intravenous (IV) antibiotic use, dry weight, serum ferritin level, saturated transferrin, parathyroid hormone level, albumin level, IV vitamin D use, and Comorbidity Index score.
48	Shunji Shiohira [66]	2016	Age, serum albumin and C-reactive protein levels, and history of CVD
49	Scott Sibbel [67]	2016	Age, race, etiology, weight, vintage, access, diabetes, congestive heart failure, cerebrovascular disease, alcohol abuse, peripheral vascular disease, and Charlson comorbidity index
50	Zijin Chen [13]	2016	age and gender
51	Rafael Perez-Garcıa [18]	2017	Age (years), CCI, VA, gender, and BMI (km/m2). ‘C-M’ denotes case-mix adjusted. This model incorporates the demographics-adjusted model and data for CRP (mg/L), hemoglobin (g/dL), Kt (L), and iron dose (mg/month)
52	Valeria Saglimbene [23]	2017	-
53	Javier Varas [68]	2017	-
54	Nada Dimkovic [69]	2017	Demographic factors, comorbidities, dialysis adequacy, and biochemical data.
55	Ko-Lin Kuo [24]	2018	Age, sex, diabetes, hypertension, dialysis adequacy (Kt/V), eGFR at the start of dialysis (MDRD), white blood cell counts, the normalized protein catabolic rate (nPCR), serum albumin, cholesterol, triglyceride, hemoglobin, ferritin, transferrin saturation, calcium, phosphate, alkaline phosphatase, intact-PTH, uric acid, and intravenous iron use
56	Toshihide Hayashi [70]	2019	Age, sex, diabetes, malignancy, eGFR, Hb, TSAT, ferritin, CRP, and intact PTH
57	Ling Sun [71]	2019	Age, hemoglobin, ferritin, TSAT, ERI, hs-CRP, pre-dialysis creatinine, albumin, and intact PTH
58	Angelo Karaboyas [72]	2019	IV iron dose
59	Shu-Ching Yeh [73]	2019	Age and sex, comorbidities such as type 2 diabetes, hypertension, congestive heart failure, left ventricular hypertrophy, cerebrovascular accident, coronary artery disease, myocardial infarction, hepatitis B, hepatitis C, and antihypertensive agents, laboratory parameters including the values of aspartate transaminase, alanine transaminase, uric acid, albumin, hematocrit, calcium, phosphorus, intact parathyroid hormone, alkaline phosphatase, and kt/V.
60	Xiangxue Lu [74]	2020	Pre-dialysis serum albumin, high-sensitivity C-reaction protein, magnesium, pre-dialysis serum ferritin, serum transferrin saturation, pre-dialysis corrected calcium, phosphorus, high-density lipoprotein, low-density lipoprotein, total cholesterol, and triglyceride
61	Sai Pan [15]	2021	Age, gender, BMI, the primary cause of ESRD, and comorbid CCVDs; type of VA, Kt/v; (iv) f hemoglobin level and iron dosage; and levels of serum albumin, serum phosphate, and serum calcium
62	Kenichi Tanaka [75]	2021	Age, sex, dialysis facility, diabetes, history of cardiovascular disease, dialysis duration, calcium, phosphorus, albumin, hemoglobin, C-reactive protein, intact parathyroid hormone, transferrin saturation, ferritin, use of angiotensin receptor blocker or angiotensin-converting enzyme inhibitor, and Kt/V
63	Takahiro Yajima [76]	2021	Age, history of cardiovascular disease, creatinine, and C-reactive protein
64	Yukio Maruyama [77]	2021	Age, sex, dialysis duration, body weight, underlying disease, and comorbid disease,
65	Marisa Roldao [78]	2022	Charlson Comorbidity Index, central venous catheter
66	Hideki Fujii [79]	2022	major adverse cardiovascular events, Cardiac events, Heart failure
67	Hyang Yun Lee [80]	2022	age, sex, and modified Charlson comorbidity index
68	Shizuka Kobayashi [81]	2022	age, dialysis history, body mass index (BMI) (median), sex, and diabetes mellitus (DM)

RETRACTED

### Evaluation of the relationship between receiving ESAs and the mortality of hemodialysis patients

Based on the results of 68 studies included in the meta-analysis of the relationship between receiving ESAs and the mortality of hemodialysis patients, it was observed that compared to the non-receiving group or group receiving the basal level of ESAs, the risk ratio (RR) of mortality in participants receiving ESAs was equal to 1.19 (95% CI: 1.16–1.23; P.value <0.001). In other words, the results of this meta-analysis show that compared to the reference group, the risk of mortality in receiving ESAs increased by 19%, which is also statistically significant (Fig 2).

**Fig 2:** Relationship between receiving ESAs and the mortality of hemodialysis patients.

### Evaluation of publication bias related to receiving ESAs and the mortality of hemodialysis patients

Evidence of publication bias was suspected upon examining the reported association between receiving ESAs and the mortality of hemodialysis patients. To investigate this, statistical tests were undertaken to evaluate potential publication bias in the reported studies (Begg’s test (p-value = 0.703) and Egger’s test (p-value≤0.001)) therefore, the results of the Egger test indicate the existence of publication bias in the study results (Fig 3). Therefore, published studies on the relationship between receiving ESAs and the mortality of hemodialysis patients are significantly associated with publication bias according to Egger’s test results, which can affect the final results of the meta-analysis [82, 83].

**Fig 3:** Evaluation of publication bias in meta-analysis studies of the relationship between receiving ESAs and the mortality of hemodialysis patients.

### Estimation of the relationship between receiving ESAs and the mortality of hemodialysis patients by considering the estimated effect size from miss studies

We tried to estimate the effect size for potentially missing studies within this meta-analysis, as depicted in Fig 4, it was estimated that five studies were missing (Fig 4). Hence, the analysis performed for this study incorporated and considered the estimated values for those potentially five missing studies. Integrating the estimated RR for the five missed studies into the analysis, showed that the RR of the relationship between receiving ESAs and the mortality of hemodialysis patients was equal to 1.13 (95% CI = 1.10–1.17; P ≤ 0.001).

**Fig 4:** Estimate the amount of effect size in the missing studies.

### Meta-regression and sensitivity analysis

In this meta-analysis, it was observed that the heterogeneity between the results of the studies is equal to 94.6%. To investigate the causes of heterogeneity, a meta-regression was performed in which variables such as the study sample size, article quality evaluation score, study design (RCTs, cross-sectional or cohort studies), the average age of participants, follow-up period, the sex ratio of study participants, place of study, and the year of the study were considered. The results of the meta-regression analysis showed that there was no significant source of heterogeneity (P>0.10).

RETRACTED

Moreover, sensitivity analysis was performed by excluding each study from the analysis one by one during each run. However, the final estimate of RR did not change significantly, which indicates the strength of the meta-analysis results (Fig 5 and Table 3).

**Fig 5:** Sensitivity analysis of the relationship between receiving ESAs and the mortality of hemodialysis patients.

**Table 3:** Sensitivity analysis of the relationship between receiving ESAs and the mortality of hemodialysis patients.

Number	Study omitted	YEAR	RR (95% CI)
1	J. Bahlmann [29]	1991	1.19 (1.16–1.23)
2	J. Möcks [19]	2000	1.20 (1.16–1.24)
3	Dennis J. Cotter [30]	2004	1.19 (1.15–1.23)
4	HAROLD I. FELDMAN [31]	2004	1.20 (1.16–1.24)
5	Deborah L. Regidor [11]	2006	1.19 (1.15–1.23)
6	Brian D. Bradbury [16]	2008	1.21 (1.17–1.25)
7	Elani Streja [32]	2008	1.15 (1.12–1.19)
8	Ryan D. Kilpatrick [33]	2008	1.20 (1.16–1.24)
9	Chang-Chyi Jenq [34]	2009	1.21 (1.17–1.26)
10	Yi Zhang [21]	2009	1.20 (1.16–1.24)
11	Huan-Cheng Chang [35]	2009	1.18 (1.15–1.22)
12	Brian D. Bradbury [20]	2009	1.20 (1.16–1.24)
13	Joseph M. Messana [36]	2009	1.19 (1.15–1.23)
14	Victor E Pollak [37]	2009	1.19 (1.15–1.23)
15	Ouhong Wang [38]	2010	1.19 (1.16–1.23)
16	Joan Fort [10]	2010	1.20 (1.17–1.24)
17	Joanne H. Lau [39]	2010	1.21 (1.16–1.25)
18	M. Alan Brookhart [17]	2010	1.21 (1.17–1.25)
19	Alexander Kainz [40]	2010	1.19 (1.15–1.23)
20	Paulo Roberto SANTOS [41]	2011	1.19 (1.15–1.23)
21	Yi Zhang [42]	2011	1.19 (1.16–1.23)
22	Eric D. Weinhandl [43]	2011	1.20 (1.16–1.24)
23	Vincenzo Panichi [44]	2011	1.19 (1.15–1.23)
24	Uyen Duong [45]	2012	1.19 (1.15–1.23)
25	Shingo Fukuma [46]	2012	1.19 (1.15–1.23)
26	Xavier Cuevas [47]	2012	1.19 (1.16–1.23)
27	Anuja Shah [48]	2012	1.20 (1.16–1.24)
28	Tetsuya Fujikawa [12]	2013	1.19 (1.15–1.23)
29	Junichi Ishigami [49]	2013	1.19 (1.15–1.23)
30	Angie Nishio [50]	2013	1.19 (1.15–1.23)
31	Wei Yang [22]	2013	1.20 (1.16–1.24)
32	Marit M Suttorp [51]	2013	1.19 (1.15–1.23)
33	Ben C. Wong [52]	2013	1.19 (1.16–1.23)
34	Nadiesda A. Costa [53]	2013	1.18 (1.14–1.22)
35	Andreas Schneider [54]	2013	1.19 (1.15–1.23)
36	Tetsuya Ogawa [55]	2014	1.19 (1.15–1.23)
37	Andreas Schneider [56]	2014	1.19 (1.15–1.23)
38	Masayuki Okazaki [57]	2014	1.19 (1.15–1.23)
39	Takahiro Kuragano [58]	2014	1.19 (1.16–1.23)
40	Vincenzo Panichi [59]	2014	1.21 (1.17–1.25)
41	Owen Kwon [60]	2015	1.19 (1.15–1.23)
42	Rieko Eriguchi [61]	2015	1.19 (1.15–1.23)
43	Myoung Nam Bae [62]	2015	1.19 (1.15–1.23)
44	Masayuki Okazaki [63]	2015	1.19 (1.15–1.23)
45	Kunitoshi Iseki [64]	2015	1.19 (1.16–1.23)
46	Elani Streja [14]	2016	1.19 (1.16–1.23)
47	Jiacong Luo [65]	2016	1.19 (1.15–1.23)
48	Shunji Shiohira [66]	2016	1.19 (1.15–1.23)
49	Scott Sibbel [67]	2016	1.20 (1.16–1.24)
50	Zijin Chen [13]	2016	1.19 (1.15–1.23)
51	Rafael Perez-Garcıa [18]	2017	1.19 (1.15–1.23)
52	Valeria Saglimbene [23]	2017	1.20 (1.16–1.23)
53	Javier Varas [68]	2017	1.19 (1.15–1.23)
54	Nada Dimkovic [69]	2017	1.19 (1.16–1.23)
55	Ko-Lin Kuo [24]	2018	1.20 (1.16–1.24)
56	Toshihide Hayashi [70]	2019	1.19 (1.15–1.23)
57	Ling Sun [71]	2019	1.20 (1.16–1.24)
58	Angelo Karaboyas [72]	2019	1.20 (1.16–1.24)
59	Shu-Ching Yeh [73]	2019	1.19 (1.16–1.23)
60	Xiangxue Lu [74]	2020	1.19 (1.15–1.23)
61	Sai Pan [15]	2021	1.19 (1.15–1.23)
62	Kenichi Tanaka [75]	2021	1.19 (1.15–1.23)
63	Takahiro Yajima [76]	2021	1.20 (1.16–1.25)
64	Yukio Maruyama [77]	2021	1.23 (1.18–1.29)
65	Marisa Roldao [78]	2022	1.19 (1.15–1.23)
66	Hideki Fujii [79]	2022	1.19 (1.15–1.23)
67	Hyang Yun Lee [80]	2022	1.19 (1.15–1.23)
68	Shizuka Kobayashi [81]	2022	1.19 (1.15–1.23)
Combined			1.19 (1.16–1.23)

RETRACTED

### Subgroup analysis

To investigate the relationship between receiving ESAs and the mortality of hemodialysis patients based on sample size, study period, study design, geographical location, the average age of participants, gender ratio (male/female), follow-up period, and the score of quality assessment, subgroup analysis was used. Based on this, it was observed that compared to the non-receiving group or group receiving basal level of ESAs, the RR of mortality in receiving ESAs group in studies with a sample size equal to or less than two thousand participants was equal to 1.25 (95% CI: 1.19–1.31; p-value≤0.001), in studies with sample size more than two thousand participants was equal to 1.16 (95% CI: 1.09–1.23; p-value≤0.001), in studies conducted in 2013 and before; was equal to 1.22 (95% CI: 1.14–1.29; p-value≤0.001), in studies conducted in 2014 and after was equal to 1.17 (95% CI: 1.12–1.22; p-value≤0.001), in the RCTs was equal to 1.06 (95% CI: 0.80–1.40; p-value = 0.701), in the cohort studies was equal to 1.20 (95% CI: 1.16–1.25; p-value≤0.001), in cross-sectional studies was equal to 1.43 (95% CI: 1.25–1.63; p-value≤0.001), in studies in American countries was equal to 1.19 (95% CI: 1.10–1.29; p-value≤0.001), in studies in Asian countries was equal to 1.15 (95% CI: 1.10–1.19; p-value≤0.001), in studies in European countries was equal to 1.18 (95% CI: 1.05–1.34; p-value = 0.007), in Austria country study was equal to 2 (95% CI: 1.47–2.72; p-value≤0.001), in international study was equal to 1.06 (95% CI: 0.87–1.29; p-value = 0.561), in studies that are in the Moderate quality score category was equal to 1.20 (95% CI: 1.09–1.32; p-value≤0.001), in articles that are in the good quality score category was equal to 1.21 (95% CI: 1.17–1.26; p-value≤0.001), in studies with an average age of 60 years and less in the participants was equal to 1.33 (95% CI: 1.15–1.55; p-value≤0.001), in the study with an average age of more than 60 years in the participants was equal to 1.13 (95% CI: 1.10–1.16; p-value≤0.001), in studies with a follow-up period of 2 years or less was equal to 1.17 (95% CI: 1.12–1.23; p-value≤0.001), in studies with a follow-up period of more than 2 years was equal to 1.23 (95% CI: 1.17–1.30; p-value≤0.001), and in studies with a gender ratio less than one was equal to 1.09 (95% CI: 1–1.19; p-value = 0.057), and in studies with a gender ratio equivalent or more than one was equal to 1.20 (95% CI: 1.16–1.24; p-value≤0.001) (Table 4).

RETRACTED

**Table 4:** Subgroup analysis in the relationship b between receiving ESAs and the mortality of hemodialysis patients.

Features of Studies		Number of studies	I^2^%	RR (95% CI)	P-value
Sample size	Equal to or less than 2000	39	87.7	1.25 (1.19–1.31)	<0.001
	More than 2000	29	97	1.16 (1.09–1.23)	<0.001
The time studying	2013 and before	35	96.6	1.22 (1.14–1.29)	<0.001
	2014 And after	33	86.4	1.17 (1.12–1.22)	<0.001
Study plan	Randomized clinical trial	5	69.1	1.06 (0.80–1.40)	0.701
	Cohort	62	94.9	1.20 (1.16–1.25)	<0.001
	Cross-sectional	1	0	1.43 (1.25–1.63)	<0.001
Geographical location	America	25	97.4	1.19 (1.10–1.29)	<0.001
	Europe	14	87.8	1.18 (1.05–1.34)	0.007
	Asia	27	86.5	1.15 (1.10–1.19)	<0.001
	Austrian	1	0	2 (1.47–2.72)	<0.001
	International	1	0	1.06 (0.87–1.29)	0.561
Quality of the article	Moderate	15	94.6	1.20 (1.09–1.32)	<0.001
	Good	53	95.4	1.21 (1.17–1.26)	<0.001
Age	60 years and less	17	93.1	1.33 (1.15–1.55)	<0.001
	More than 60 years	48	90.3	1.13 (1.10–1.16)	<0.001
Study follow-up period	2 years and less	40	95.9	1.17 (1.12–1.23)	<0.001
	More than 2 years	27	89.8	1.23 (1.17–1.30)	<0.001
Gender ratio (male/female)	Less than 1	8	86.1	1.09 (1–1.19)	0.057
	More than 1	56	91.4	1.20 (1.16–1.24)	<0.001

## Discussion

This systematic review and meta-analysis were conducted to review the relationship between receiving ESAs and the risk of mortality in hemodialysis patients. In this study, 68 articles were included in the meta-analysis, and the final estimate of the RR indicated that compared to the non-receiving group or group receiving the basal level of ESAs, the RR of mortality in receiving ESAs was equal to 1.19 (95% CI: 1.16–1.23; P.value <0.001). In this regard, it should be mentioned that the results of the present study are align with the results of most investigators’ studies regarding the relationship between receiving ESAs and mortality in hemodialysis patients. After several clinical trial studies found that patients randomized to groups with higher HB target levels had higher mortality rates [6, 7], the US Food and Drug Administration recommended a more conservative ESA dosing regimen for the treatment of patients with chronic kidney disease [84]. In a study conducted by Streja E et al. to determine the relationship between ESAs and mortality in hemodialysis patients, it was observed that compared to an ESA dose of <6000U/week, the adjusted odds ratio of mortality for an ESA dose of 6000 to <12000 U/week was equal to 1.02 (95% CI: 0.94–1.10), for ESA dose of 12000 to <18000 U/week was equal to 1.08 (95% CI: 1.00–1.18), for ESA dose of 18000 to <24000 U/week was equal to 1.17 (95% CI: 1.06–1.28), for ESA dose of 24000 to <30000 U/week was equal to 1.27 (95% CI: 1.15–1.41), and for ESA dose ≥30000U/week was equal to 1.52 (95% CI: 1.37–1.69) [14]. In this study, it was observed that the risk of mortality increases with the increase in the dose of ESA. Similarly, in the study of Regidor DL et al., which was conducted in 2006 to investigate the relationship between hemoglobin changes and ESAs with survival in hemodialysis patients, it was observed that the decrease in hemoglobin followed by the need for higher doses of ESA in hemodialysis patients is associated with an increase in the mortality of these patients [11]. Likewise, in the study conducted by Bradbury BD et al. in 2008, a statistically significant relationship was observed between receiving ESAs and increased mortality, so that for each EPO unit dose increase, the relative risk of mortality increased by 1.31 (95% CI:1.26–1.36) [16]. In this regard, a study entitled " Relationship between epoetin alfa dose and mortality: findings from a marginal structural model " were conducted on 27,791 hemodialysis patients by Wang O et al. the findings of this study showed that in hemodialysis patients, relative to the group received ESAs with dose less than 14000 U/week, the RR of mortality in the group receiving 14001–27000 U/week is equal to 1.07 (0.91-1-33), in the group receiving 27,001–49,000 U/week was equal to 1.21 (1-1-53) and in the group receiving more than 49,001 U/week, it was equal to 1.39 (1-08-1-91) [38].

RETRACTED

The results of the research of Santos PR et al., also showed that compared to patients receiving the usual dose of EPO, the RR of mortality in patients who use high doses of EPO is equal to 2.96 (95% CI:1.13–7.77) [41]. Furthermore, in a cohort study conducted with Nishio A et al., on 606 hemodialysis patients observed that higher ESA doses were associated with a significant increase in the risk of all-cause mortality. So that for each 100 μg increase in the total weekly dose of darbepoetin alfa, risk of mortality 9% increased [50]. In addition, Perez-Garcıa et al., observed that ESA doses greater than 8000 units per week were associated with an increased risk of all-cause mortality and hospitalization in HD patients [18]. Similarly, Pan et al., also observed that ESA dose more than 10,000 units per week in the first 3 months for Chinese hemodialysis patients was associated with an increased risk of all-cause mortality [15]. In the study of Kainz A et al., it was observed that, if the hemoglobin concentration was maintained stably in the range between 10 and 12 g/dL, compared to the group that received less than 16,000 U/week of ESAs, the RR of mortality in the group that received more than 16,000 U/week is equal to 1.3 (95% CI:1.02–1.64) [40]. In the subgroup analysis on the RCTs studies considered in this study, observed that compared to the group receiving the basal level of ESAs, the RR of overall mortality in patients receiving ESAs was equal to 1.06 (95% CI:0.80–1.40), although this increase is not statistically significant. In a clinical trial study conducted by Joanne H. Lau et al., it was observed that increasing the level of ESA intake in hemodialysis patients leads to an increased risk of mortality, so for every 1000-unit increase in ESA dose, the adjusted HR was 1.12 (95% CI:1.01–1.24) [39]. Similarly, in another clinical trial study conducted in this field on hemodialysis patients with type 2 diabetes, it was observed that patients with ESA resistance had significantly higher mortality as compared to non-resistant patients in the first year of follow-up (HR 1.77, 95% CI: 1.23–2.54) [54]. However, in some studies, a statistically significant relationship between the increased dose of ESAs and mortality has not been observed. For example, in the study of Bradbury BD et al., in 2009, no statistically significant relationship was observed between the dose of ESAs and the risk of mortality [20]. Similarly, in a number of clinical trial studies conducted in this field, a statistically significant relationship between receiving or increasing the level of erythropoietin and the risk of mortality in hemodialysis patients hasn’t been observed [23, 29, 33].

This study is one of the most comprehensive studies that has been conducted so far in the field of investigating the relationship between ESAs and mortality in hemodialysis patients; because it includes more and more up-to-date studies, and tried to calculate the effect of missing studies and considers it in estimating the final effect size of the study, also in this study, subgroup analysis, meta-regression, and sensitivity analysis were performed, which help in identifying the root of heterogeneity in the results of the studies used in this analysis. It has been tried to present the results of the study in more detail with the use of the results of subgroup analysis. However, this study does not helpful to determine the best ESAs dose for use in hemodialysis patients. In addition, it should be pointed out that most of the studies included in this meta-analysis are observational studies (cohort and cross-sectional), so it is necessary to design and implement more studies with RCTs structure in the field of assessing the relationship between receiving ESAs and mortality in hemodialysis patients. Considering that in the meta-analysis of clinical trial studies, although a 6% increase in the risk of mortality was observed, this increase is not statistically significant. Therefore, conducting clinical trial studies with a larger sample size in this field can be very helpful, because the sample size of clinical trial studies conducted in the field of investigating the relationship between erythropoietin intake and mortality risk is equal to 2275 patients. Clearly, this number of samples is not suitable for obtaining a causal conclusion.

RETRACTED

The need for higher ESA doses may reflect underlying pathologies that increase mortality risk. Comorbidity indices could not be evaluated since we only had access to aggregated study-level data rather than individual participant data. However, S1 Table S1 File details the prevalence of underlying diseases among subjects in each study. A higher comorbidity burden could associate with both increased mortality and higher ESA requirements. These limitations restrict causal interpretations of the findings. Specifically, we cannot infer a causal relationship between high-dose ESA and increased mortality in hemodialysis patients based on this meta-analysis alone. Nonetheless, the significant statistical association underscores the need for further mechanistic research and investigations into optimal ESA dosing in this population.

## Conclusion

In summary, the results of this study show that the use of erythropoietin is associated with a 20% increase in the risk of overall mortality in hemodialysis patients. The results of this study support the current conservative ESA dosing regimen, which aims to strike a balance between the potential harms of higher doses of ESAs and the anemia-correcting benefits of receiving them. However, more studies are necessary, especially with RCTs or cohort design, to create an ideal ESA dose algorithm in hemodialysis patients, as well as biological studies to understand the complex pathophysiological relationship between ESA dose and mortality.

RETRACTED

## Supporting information

S1 File (PDF)
